The article "Named Entity Recognition of Medical Text Based on the Deep Neural Network" was retracted in 2023. Reasons: signs of a paper mill; suspected computer-generated content; unreliable results or conclusions; concerns about the data.

# Named Entity Recognition of Medical Text Based on the Deep Neural Network

**DOI:** 10.1155/2022/3990563

**Published:** 2022-03-07

**Authors:** Tianjiao Yang, Ying He, Ning Yang

**Affiliations:** ^1^College of Electronic Information, Qingdao University, Qingdao, Shandong 266071, China; ^2^Qingdao Lanzhi Modern Service Industry Digital Engineering Technology Research Center, Qingdao, Shandong 266071, China

## Abstract

Medical text data records detailed clinical data; named entity recognition is the basis of text information processing and an important part of mining valuable information in medical texts. The named entity recognition technology can accurately identify the information needed in medical texts and help medical staff make clinical decision-making, evidence-based medicine, and epidemic disease monitoring. This paper proposes a hybrid neural network medical text named entity recognition model. First, a coding method based on a fully self-attentive mechanism is proposed. The vector representation of each word is related to the entire sentence through the attention mechanism. It determines the weight distribution by scoring the characters or words in all positions and obtains the position information in the sentence that needs the most attention. The encoding vector at each position is integrated with the context information of full sentence, which solves the ambiguity problem. Second, a multivariate convolutional decoding method is proposed. This method can effectively pay attention to the characteristics of medical text named entity recognition in the decoding process. It uses two-dimensional convolutional decoding to associate the current position word with surrounding words to improve decoding efficiency while extracting features from the logic of the preceding and following words. Using the same number of convolution kernels as the entity category, it can effectively extract effective features from the label dimension. Besides, according to the characteristics of the named entity recognition task, a special mixed loss is designed. The experimental results verify that the proposed method is effective, and it is improved compared with some existing medical text named entity recognition methods.

## 1. Introduction

With the vigorous development of artificial intelligence, natural language processing (NLP) has always been a research hotspot. The ever-increasing performance of computing devices and the ever-developing algorithms have resulted in the emergence of a large number of excellent new algorithms for natural language processing on a large number of tasks. For the ever-changing Internet industry, how to combine the existing massive text data and natural language processing technology to mine the valuable data information in the massive text is a very challenging task. Artificial intelligence technology is entering all aspects of modern society and is gradually playing an irreplaceable role in all walks of life, and natural language processing technology is changing people's lives [1–5].

When it comes to proper names and phrases, named entity identification is the most important part of the process. There are a variety of downstream activities that rely on named entity identification as a building block, including information extraction, knowledge graphs, automated question answering, and machine translation. Named entities in nonspecific domain text data generally refer to specific referring entities. In specific field data such as medical data, named entities are mostly entities such as genes, diseases, and drugs. Named entity recognition system extracts entities from unstructured unlabeled text and performs sequence labeling tasks according to different standard rules [6–10].

At present, medicine is developing rapidly, and a large amount of medical information exists in various forms of text in an unstructured form. It can provide a large amount of professional data and knowledge for scientific research and teaching. With the popularization of informatization, a large amount of medical data has been accumulated in various business systems of hospitals, and these data have the characteristics of being heterogeneous, distributed, fragmented, and so on. The use of computers to process and analyze huge amounts of medical text data requires further research and development of natural language processing technologies corresponding to medical texts. The mining of medical text data is a cross-discipline of computer and medicine. It often involves machine learning, deep learning, artificial intelligence, and other fields in the field of computer science. In order to effectively analyze and mine these data through existing analysis methods, medical data needs to be structured. Through the use of natural language processing, named entity recognition of text data in the medical field will lay the foundation for the structured representation of data. Using effective computer algorithms and improving the accuracy of algorithm recognition is an indispensable link in medical text data mining. Medical text named entity recognition aims to identify specific text blocks in specific medical texts. It is extremely important in extraction of disease treatment relationship, gene function recognition, and semantic relationship extraction of molecular biology ontology concepts. Different from traditional named entity recognition, the medical field pays more attention to entities such as symptoms, organs, treatment methods, drugs, and diseases. However, due to the lack of standard naming methods in medical research, few models can achieve very satisfactory results. So medical text named entity recognition is still a very difficult issue [11–15].

In order to solve the problems existing in medical text entity recognition, this paper conducts corresponding research based on deep neural network. This work designs a medical text named entity recognition model with hybrid neural network. According to the characteristics of word ambiguity and structural complexity of medical text, a fully self-attentive coding mechanism is designed, which integrates contextual information into the coding of each word. It eliminates the problem of the disappearance of the long-distance transmission gradient caused by the use of time series model coding. At the decoding end, a multivariate convolutional decoding method is proposed to allow it to fully capture information in different feature dimensions. In addition, according to the characteristics of the named entity recognition task, a special mixed loss is designed, so that the convolution kernel can perform feature modeling for each label category.

## 2. Related Work

The method based on rules and dictionaries was mainly based on artificially defined rules and pattern matching to generate dictionaries and extract medical entities from existing medical dictionaries. Literature [16] used custom vocabulary and grammatical rules to identify medical knowledge in X-ray reports. Literature [17] used medical dictionaries to extract medical concepts from clinical texts and achieved good results. Although the method based on dictionaries and rules was simple to implement, the accuracy was closely related to the manually formulated rules and the quality of constructing medical dictionaries. It not only required researchers to fully analyze the corpus but also needed to have experience in the medical field. In addition, due to the rapid development of medical research, it was becoming more and more difficult to construct high-quality medical dictionaries. Normally, most dictionaries could not cope with large-scale and diversified medical data. In addition, the effect of this method was greatly reduced in practical applications due to the irregularities in the naming of entities in medical texts.

Methods based on machine learning consider it was a sequence labeling issue. The corresponding label for each character in the input sequence was predicted and the entity in the sentence was identified according to the label sequence. Literature [18] used a semi-Markov model to label conceptual entities in sequence. By adopting four tags and introducing concept mapping features and context features, it had obtained a better entity recognition effect. Literature [19] combined support vector machines with conditional random fields to identify entities in electronic medical records. Literature [20] used statistical models to extract concepts from clinical texts from multiple data sources and used BioTagger-GM to train the model to learn labels. Literature [21] used SVM and maximum entropy model, combined with rules to identify named entities in electronic medical records. These methods could achieve good and stable results in entity recognition tasks but to a large extent depend on artificially formulated features. This had limited the scope of application of this method.

Named entity recognition methods based on deep learning were used in entity extraction tasks. Literature [22] introduced the attention mechanism to recognize chemically named entities based on the deep learning model, which solved the problem of label inconsistency. Literature [23] trained two-way language model vectors on massive unlabeled corpus and added feature vectors to the original two-way recurrent neural network and CRF model for semisupervised sequence labeling. Literature [24] combined Bi-RNN and CRF and introduced n-gram features to identify five types of entities in Chinese clinical electronic medical records. Literature [25] proposed a transfer bidirectional recurrent neural network, which automatically extracted medical concepts such as diseases and treatments from Chinese electronic medical records. Literature [26] used the minimum feature engineering method and proposed two deep neural networks. Unsupervised learning was used to generate word vectors from a large number of unlabeled corpora to perform named entity recognition tasks. This method was superior to the existing CRF model, which shows the effectiveness of unsupervised learning. In order to establish high-precision drug entity recognition and clinical concept extraction, literature [27] combined the bidirectional LSTM with the CRF model to form BiLSTM-CRF model and used the dataset in the health field to train to get richer and professional word vectors, avoiding the manual construction of features. Literature [28] used large-scale unlabeled corpus to learn multiple representations of entity categories and mined the semantic relationship between clinical medical entities and text words. Literature [29] proposed a model combining speech and self-matching attention mechanism. This improved the accuracy and performs well in clinical entity recognition. Literature [30] proposed a deep residual network with attention mechanism to extract medical information. It enhanced the recognition characteristics of different types of entities by combining the attention mechanism of character position. Literature [31] introduced word level information on the basis of the BiLSTM model. Different features based on dictionaries were combined to identify entities such as diseases and drugs in Chinese electronic medical records and obtain better recognition results. Compared with machine learning methods, methods based on deep learning could automatically learn features. They did not require manual definition, had strong generalization ability, and could better analyze entity performance.

## 3. Method

To effectively identify medical text entities, this paper proposes a hybrid neural network (HNN) as illustrated in Figure 1. FSAE refers to fully self-attentive encoder. MCD refers to multivariate convolutional decoder. The rest of this section will explain the composition of the network in detail.

### 3.1. Fully Self-Attentive Encoder

This section focuses on the characteristics for medical text named entity recognition tasks, such as the ambiguity of words and characters and the disappearance of the long-distance transmission gradient of the temporal neural network framework. A fully self-attentive coding model is proposed to extract features for medical text named entity recognition tasks. It can directly transmit information regardless of the distance between words or characters in a sentence, and there is no restriction on the characteristics of time series data.

#### 3.1.1. Motivation

The existing named entity recognition algorithms basically treat sentences as time series data. The reason for this is based on the assumption that the reading habit is to read sequentially in a fixed direction, which is in line with the characteristics of time series data. Text-named entity recognition model with deep learning that has achieved good result uses time series model as the main framework, and the sentences are input into the model. Compared to RNN, the network structure of LSTM adds input gates, forget gates, and output gates. This makes it possible to decide which information needs to be forgotten and which information needs to be passed on to the next time step. This solves the problem of explosion or disappearance of the information gradient caused by the long-distance sequence of RNN to a certain extent. But, for the task of naming entities in medical texts, there are still shortcomings. The vocabulary of medical texts is more polysemous, and, generally, only by reading the whole sentence can we clearly judge the meaning of some words in the sentence.

How to make each word better integrate its context information when encoding a sentence has become the key to the effectiveness of the task of medical text named entity recognition. In addition, time series neural network models such as LSTM and GRU have very high requirements for hardware. Their structure determines that four fully connected layers are required in the core of each LSTM. If the time step of LSTM is very long and the number of layers is very deep, then the volume of the model will be quite huge; and because of the time sequence of LSTM, it cannot accelerate the calculation in parallel, which will cause medical text named entity recognition to use LSTM and other time series models as framework training on any dataset, which is a huge test for the hardware.

Therefore, this paper proposes a fully self-attentive encoder to replace the above-mentioned temporal model to model the corpus. The fully self-attentive mechanism pays attention to the words in all positions in the sentence when extracting the characteristics of the characters in each position and scores these words according to the degree of influence on the current word. In this way, the feature vector of each word will be fused with contextual information that is valid for it.

The fully self-attentive encoder does not have the timing characteristics of the time series model, so it cannot distinguish the sequence of words in the sentence. However, this article does not use additional coding information to increase the sequence characteristics of words, mainly based on the assumptions made by people's habits in fast reading in daily life. Combined with the characteristics of named entity recognition for medical text, the task does not require natural language processing tasks such as translation and question answering, and the semantics of the entire sentence can be extracted very accurately and completely. Instead, it only needs to extract the key entity words and judge their categories. Aiming at this characteristic, there is only a need to perform effective feature extraction on the part of the entity and pay attention to other key words in the sentence which affect its word meaning. In this way, it is possible to avoid the complexity of the model that the time series model needs to extract the semantics of the entire sentence, as well as the interference caused by the important local feature extraction part. In addition, the operation of the fully self-attentive mechanism is based on matrix operations, which determines that it can accelerate calculations in parallel through GPUs.

#### 3.1.2. Structure

The fully self-attentive encoder does not use a timing model. Instead, in the encoding process of each position, all the words or word embedding vectors in the sentence are input into the self-attentive mechanism to calculate the weight assigned to each position. Finally, the code of the current position is obtained. The structure of the fully self-attentive coding model is shown in Figure 2.

(1) $$\begin{array}{c} E=\left[e_{1},e_{2},e_{3},\ldots ,e_{n}\right], \end{array}$$

where *n* is the length for input and *e*_*i*_ is the word vector after embedding.

The word vector matrix *E* is input to the self-attentive mechanism *n* times, and the output of the *i*-th input is

(2) $$\begin{array}{c} a_{i}=\text{Att}\left(e_{i};E\right). \end{array}$$

There is no priority when inputting, and input operations can be performed at the same time. Splice the full attention code *a*_*i*_ obtained each time into the final output of the fully self-attentive code:

(3) $$\begin{array}{c} A=\left[a_{1},a_{2},a_{3},\ldots ,a_{n}\right]. \end{array}$$

#### 3.1.3. Working Mechanism

The self-attentive mechanism encodes each word, which can effectively extract contextual information features into the current word hiding vector. This makes it pay attention to the position in the sentence related to the classification of its named entity.

From a macro perspective, the recurrent neural network encodes the words in an input sentence by combining all the previously processed information with the currently encoded words to generate a target vector. The self-attentive mechanism for word encoding will directly focus on all words in the sentence and assign weights according to the influence of these words on the current encoded word. Theoretically, if certain words are not related to the named entity classification of the current word, the assigned weight can be infinitely close to zero.

The realization of the self-attentive mechanism is viewed from a micro perspective. First, the self-attentive mechanism generates three vectors for each word or word embedding vector, the query vector, the key vector, and the value vector. These three vectors are the dot product of the embedding vector and three custom parameter matrices. The three parameter matrices are also optimized through top-down neural network training. After getting the three vectors, you need to use them to score all the words in the sentence. First, use the query vector of the currently encoded word and the key vector of all words including itself to do a dot product. The value obtained is the influence of all words in the sentence on the word. The larger the value is, the more important the word is to the currently encoded word. Then use the softmax function to normalize the scores so that scores obtained are all positive and the sum of all the scores is equal to 1. Here, the softmax score of each word is equivalent to its contribution to the word encoding at the current position. Finally, multiply the value vector of each word by its corresponding softmax score, and the final vector of the sum of the vector values is the self-attentive vector of the word at the current position. The goal of the model here is to weaken words that are not related to the current word as much as possible, and the value of softmax is as small as possible. It can be seen that the word hidden vector encoded in this way fully integrates the context information needed by oneself and can effectively pay attention to the position of the word related to the entity recognition classification. Moreover, it can prevent the weakening and disappearing of information transmission caused by too long sentences and too far apart words.

The output matrix formula of the fully self-attentive coding layer of the model can be expressed as

(4) $$\begin{array}{c} A=\text{soft }\max\left(W_{q}W_{k}^{T}W_{v}\right), \end{array}$$

where *W*_*q*_, *W*_*k*_, and *W*_*v*_ are three parameter matrixes.

### 3.2. Multivariate Convolutional Decoder

This section proposes a multivariate convolutional decoding framework to solve the problem of entity nesting that often occurs in medical text named entities. At the same time, it enables each word to be associated with the grammar and word meaning information of adjacent words in the decoding process. In addition, multiple filters are used in the convolution process to decode each tag category separately to optimize the feature extraction in the tag dimension as much as possible.

#### 3.2.1. Motivation

At present, named entity recognition tasks mainly use CRF (Conditional Random Fields) as the decoding layer of the model. The main reason why CRF are used for decoding is that they can incorporate dependencies in named entity tags. The parameter of CRF is *P* ∈ ℝ^(*t*+2)×(*t*+2)^, where *t* is the number of tags in the current named entity recognition, and *P*_*ij*_ represents the transfer score from the *i*-th tag to the *j*-th tag. Therefore, current label for the sentence is judged based on the position that has already been marked. The score of the input sentence *f*=[*f*_1_, *f*_2_,…, *f*_*n*_] with the output label *g*=[*g*_1_, *g*_2_,…, *g*_*n*_] is

(5) $$\begin{array}{c} \text{score}\left(f,g\right)=\sum_{i=1}^{n}h_{i,g_{i}}+\sum_{i=1}^{n+1}P_{g_{i-1},g_{i}}, \end{array}$$

where *h*_*i*_ is the hidden vector output from the previous layer such as Bi-LSTM. The scoring for entire sequence is composed of the sum of the scores of each part, and the scoring of each part is composed of two parts. The left part is the feature vector output by the model coding layer, and the right part is the CRF transition matrix.

When only considering the sequence of interactions between two consecutive tags, CRF model decoding usually uses the Viterbi algorithm to find the tag sequence. For NLP tasks, the amount of data in the corpus is huge and the data dimension is high, and the use of Viterbi algorithm will be very complicated. Secondly, CRF is similar to LSTM. It needs to calculate the current time series label based on the decoding result of the previous time series, so it cannot accelerate the operation in parallel. Judging from the fully self-attentive coding model proposed in this paper, it does not use sequence labeling models such as LSTM. Therefore, it is not suitable to directly use the Viterbi algorithm in the field of dynamic programming. At the same time, based on the assumptions put forward in this article, named entity recognition task does not need to understand and model the semantics of the whole sentence. In the same way, for the dependencies between sequences, there is no need to dynamically plan the labels of the entire sentence but only need to perform association modeling for a part of adjacent positions each time. In addition, CRF only performs feature extraction modeling for the front and back dependencies of tags during decoding. It does not perform feature extraction on the information contained in other underlying coding vectors. This article hopes to decode the model in a deeper dimension based on the characteristics of named entity recognition while decoding.

Therefore, this work proposes a decoding method with multivariate convolution, which uses the convolution operation on the adjacent *n* hidden vectors to replace the CRF to model the dependency of the label before and after it. In the convolution, this paper uses the same convolution kernel with the same number of tags as the named entity recognition task, constructs multiple feature maps, and then uses the multilayer perceptron and softmax function. This enables the decoding process to perform feature extraction in the dimension of the tag type, enlarge the feature of the tag at the current position, and weaken the features of other tag classifications.

#### 3.2.2. Structure

The framework of the multivariate convolutional decoder concatenates each position with its adjacent *k* − 1 position vectors and then performs a convolution operation on the resulting matrix. The framework of the MCD is shown in Figure 3.

The input of multivariate convolutional decoding layer is the output from the last neural network. In this article, the word embedding is coded for each word, and the sequence *A*=[*a*_1_, *a*_2_, *a*_3_,…, *a*_*n*_] is generated by the self-attentive mechanism.

In the multivariate convolutional decoding, each self-attention vector *a*_*i*_ is concatenated with *k* − 1 vectors before and after itself into a matrix with itself as the center:

(6) $$\begin{array}{c} A_{i}=\left[a_{1-k+1},\ldots ,a_{i},\ldots ,a_{i+k-1}\right]. \end{array}$$

Each matrix is convolutionally decoded through convolutional layers. Each filter generates a vector of 1 × *k*, and then each filter generates a vector *c*_*i*_ end to end. The formula for generating matrices for all *A*_*i*_ through convolution is

(7) $$\begin{array}{c} C=\text{Concat}\left(\text{Conv}\left(\left[A_{1},\ldots ,A_{n}\right]\right)\right). \end{array}$$

After each vector *c*_*i*_ is generated by MLP, it is normalized using the softmax function, and finally its corresponding label is output.

#### 3.2.3. Working Mechanism

This work uses multivariate convolution method to decode the output vector of the coding layer. The purpose is to associate and jointly decode the surroundings of the current decoding position during decoding based on the characteristics of named entity recognition of medical text. This solves problem for named entity nesting and label dependency. For the output of the previous layer, each dimension can be individually connected to multiple fully connected layers and finally converted into a vector and then decoded using the softmax function. Using a multilayer perceptron to directly decode a single hidden vector can extract the features of words or characters extracted by itself to the greatest extent. However, it does not combine the vectors of the front and back positions so that it cannot extract the remaining position information related to the named entity at the current position.

Therefore, the model in this article uses a convolution operation to decode the encoding layer. Convolutional neural networks are not like a fully connected layer in a multilayer perceptron, which connects neurons to each other. However, it can make the text sentence problem in natural language processing analogous to the solution of the image problem and perform regionalized decoding to extract the characteristics of a segment of adjacent words in the sentence. Generally, when a convolutional neural network is used in a natural language processing task, it convolves a matrix composed of vectors of the entire sentence, so as to extract the semantics of the entire sentence sequence or the required features in classification tasks such as sentiment. This paper believes that the task of medical text named entity recognition does not need to convolve the entire sequence every time in the decoding stage. First of all, the full self-attentive coding framework used in the previous section has already performed fusion feature extraction for the entire sentence. If feature extraction is performed on the entire sequence in the decoding layer, there will be redundancy. Secondly, for some characteristics of named entity recognition, when decoding, focusing on the adjacent words to determine the type of label will greatly improve the accuracy.

The multivariate convolution decoder designed in this paper takes the current position vector as the center, and the matrix formed by splicing *k* − 1 vectors before and after it is the convolution range for two-dimensional convolution. If there are less than *k* − 1 vectors before and after the current position vector, padding will be filled. The convolutional neural network used in this article does not use a pooling layer after convolution but stitches all the convolution results together as the input of the next layer. Because, as a convolutional neural network for named entity recognition, the result of each convolution reflects the characteristics of the current position and part of the adjacent position, it should be reserved as effective information for the lower layer to extract. In order to reflect the characteristics of the named entity recognition task, for the classification of multiple entity categories, this paper uses multiple filters to convolve the sequence matrix. The number of filters is the number of entity tag categories. The convolution results of each filter are first spliced into a one-dimensional vector. The result of the convolutional layer is the same as that of the multilayer perceptron, and the final output is a 1 × *t* one-dimensional vector, where *t* is the number of named entity tag categories. Finally, connect the softmax function for normalization.

### 3.3. Mixed Loss

The task of medical text named entity recognition needs to distinguish each word (character) in the input sequence as an accurate entity classification or nonentity. Therefore, most of the named entity recognition is a multiclassification task. In view of this feature, the number of filters of the convolutional neural network in the multivariate convolutional decoding layer is set to the number of tag types of the current named entity recognition task. In this way, each coding vector can extract the corresponding characteristics in all the dimensions of the label category. Theoretically, it is hoped that each set filter can correspond to the feature extraction of a tag category, and the features extracted by the filter corresponding to the current word classification should be given a higher weight. Conversely, the features extracted by other filters should be weighted as low as possible.

Therefore, the model needs to be modified during training. The filter of convolutional neural network can extract corresponding label features, and it can make the extracted features distinguish whether the corresponding tag is the tag type of the current location. Therefore, this paper proposes a mixed loss strategy. It uses two classifications and multiple classifications in named entity recognition at the same time, and the multitask loss function is used to train the model to achieve the purpose of improving the model's ability to extract features in the label category dimension. This effectively improves the accuracy of model entity recognition.

The decoding model proposed in this paper is designed to be able to use multiple filters in the feature extraction layer of the convolutional neural network for convolution operations. This allows each filter to extract the features of the encoding vector in a tag category in a targeted manner. In order to achieve this goal, this article is different from the inference model in the training model, which only trains the multiclassification task with the final desired result. However, multiple binary classification tasks are added to the convolutional neural network layer during decoding, allowing it to judge whether the word or character at the current decoding position is in each label category. The specific implementation process is shown in Figure 4.

At the decoder layer, this article sets the number of filters consistent with the number of tag types in the dataset. Each filter will perform a multivariate convolution operation on the current word or character encoding position to obtain a one-dimensional feature vector. For *t* filters, *t* feature vectors will be obtained. In order to make the feature vector results obtained by convolution of each filter represent the dimensional features of a specific label type, in the training phase, the model performs a two-classification task training on each feature vector. Each vector in turn corresponds to a label in the set. Each feature vector passes through a multilayer perceptron, and the last output of the perceptron is two nerves, and then the softmax normalization operation is performed on it.

The cross-entropy loss function formula for a filter extraction feature result of a single sample is

(8) $$\begin{array}{c} L_{1}=-\sum p\left(i\right)\log\left(q\left(g\left(f\left(i\right)\right)\right)\right), \end{array}$$

where *p* is the true label value of the sample and *q* is the actual output of the model.

For the coding vector of the word or character at the current position, the training model performs two classifications in addition to each label category. The feature vector generated by each filter must also be spliced to complete the multiclassification task of predicting the type of label. This part is consistent with the principle of the inference model, and its loss function formula is

(9) $$\begin{array}{c} L_{2}=-\sum p\left(C\right)\log\left(q\left(g\left(C\right)\right)\right), \end{array}$$

where *C*=[*f*_1_, *f*_2_,…, *f*_*n*_]. The mixed loss function of the multiclassification task and the two-classification task is

(10) $$\begin{array}{c} L=L_{1}+L_{2}. \end{array}$$

## 4. Experiment and Discussion

### 4.1. Dataset and Metric

This article uses a self-made medical text dataset, which is a dataset for named entity recognition and evaluation tasks for electronic medical records. It is mainly composed of hospitalized medical records, including the first page of hospitalized medical records, admission records, course records, and pathological data. The dataset contains five entity types: Anatomy, Symptom, Independent, Drugs, and Operation. The statistical results of the entities are shown in Table 1. Among them, the training set includes 800 current medical history documents, and the test set includes 400 current medical history documents.

Medical text named entity recognition needs to judge the entity boundary and entity type. This paper uses the accurate evaluation method, and only when the boundary and type of the entity are consistent with the true label value is the entity recognition considered correct. At the same time, three evaluation indicators are used to quantitatively analyze the effect of the model, namely, precision, recall, and F1 score.

### 4.2. Comparison with Other Methods

To verify the effectiveness of our designed model, this section compares our method with other methods including CPM [32], JIC [33], FSCBR [34], and MDD [35]. Experimental result is illustrated in Table 2.

Obviously, compared with the listed methods, our method can obtain the optimal performance. Compared to the best method MDD, our model can obtain 0.9%, 1.4%, and 0.8% gains on precision, recall, and F1 score. This demonstrates the efficiency of our method.

### 4.3. Evaluation on Network Convergence

In the neural network, the convergence of the model is an important evaluation metric for evaluating network performance. If the network cannot converge, subsequent predictions are meaningless. Therefore, this paper compares the training loss and the testing performance. Experimental result is illustrated in Figure 5.

With the training progresses continuing, the loss of the network gradually decreases, and the test performance of the network gradually increases. When the training epoch is 100, the loss no longer drops, and the test performance no longer rises. The final three performance indicators are 0.924, 0.907, and 0.915. This shows that the network has reached a state of convergence, and the designed network can finally converge and make stable and efficient predictions.

### 4.4. Evaluation on the Fully Self-Attentive Encoder

In this work, a fully self-attentive encoder is proposed to replace the time series modeling encoder. To verify the effectiveness of this strategy, we compare the encoders using timing model with FSAE. The result is illustrated in Figure 6.

Obviously, when using LSTM or Bi-LSTM to replace the FSAE module proposed in this article, the three performance indicators all have different degrees of decline. This shows that the fully self-attentive mechanism, a nonsequential coding model, can model medical text named entity recognition more effectively.

### 4.5. Evaluation on the Multivariate Convolutional Decoder

In this work, a multivariate convolutional decoder is proposed to replace the CRF encoder. To verify the effectiveness of this strategy, we compare the model using CRF encoders with FSAE. The result is shown in Figure 7.

Obviously, when using CRF to replace the MCD module proposed in this article, the three performance indicators all have different degrees of decline. This shows that the multivariate convolutional decoder can model medical text named entity recognition more effectively.

### 4.6. Evaluation on Mixed Loss

In this work, a mixed loss consisting of two-classification loss and multiclassification loss is proposed to optimize the network. The training model is different from the inference model, which only trains the multiclassification task with the final desired result. However, during the decoding process, multiple two-classification tasks are added to the capacity neural network layer, allowing it to decide whether the word or character at the current decoding position is of this class on each label class. To verify the effectiveness, we compare the network only using multiclassification loss with mixed loss. The result is shown in Figure 8.

Obviously, when using the single multiclassification loss to replace the mixed loss proposed in this article, the three performance indicators all have different degrees of decline. This shows that the mixed loss can optimize the network more effectively and guide the network to extract more discriminate features for medical text named entity recognition.

## 5. Conclusion

In order to meet the challenge, this paper analyzed some existing medical text named entity recognition models and pointed out their possible shortcomings and proposed a hybrid neural network model. This model improves the performance of medical text named entity recognition. First, this work proposes a coding model based on full self-attention. The words in medical text are more polysemous, and the meanings of some words in the sentence can be clearly judged by reading the whole sentence. Therefore, this paper proposes a fully self-attentive model to replace the temporal model to model the corpus. The fully self-attentive mechanism pays attention to the words in all positions in the sentence when extracting the features of the words in each position. These words are scored according to the degree of influence on the current word. In this way, the feature vector of each word will incorporate contextual information. Second, this paper proposes a decoding method based on multivariate convolution. It uses convolution operation on adjacent hidden vectors instead of CRF to model the dependency relationship between labels. In the convolution, this paper uses the same number of convolution kernels as the number of tags for the named entity recognition task. It constructs multiple feature maps and then uses multilayer perceptron and softmax function. Even the decoding can perform feature extraction in the dimension of the full label, amplify the features of the label at the current position, and weaken the features of other label classifications. Third, multiple binary classification tasks are added to the convolutional neural network layer when the training model is decoded. A large number of experiments verify the effectiveness and reliability of our method.

## Figures and Tables

**Figure 1:** The structure of the HNN.

**Figure 2:** The structure of FSAE. The model input is the word vector after word embedding.

**Figure 3:** The structure of MCD.

**Figure 4:** Model multitask training mechanism.

**Figure 5:** The training loss and test performance.

**Figure 6:** Evaluation on the fully self-attentive encoder.

**Figure 7:** Evaluation on the multivariate convolutional decoder.

**Figure 8:** Evaluation on mixed loss.

**Table 1:** Dataset entity statistical result.

Item	Document	Anatomy	Symptom	Independent	Drugs	Operation
Train	800	7534	3019	3407	1658	1427
Test	400	4083	1482	1632	915	748

**Table 2:** Comparison with other methods.

Method	Precision	Recall	F1
CPM	0.873	0.848	0.861
JIC	0.892	0.871	0.882
FSCBR	0.906	0.885	0.894
MDD	0.915	0.893	0.907
Ours	0.924	0.907	0.915

## Data Availability

The datasets used during the current study are available from the corresponding author upon reasonable request.

## References

[1] Wolf T., Chaumond J., Debut L. Transformers: state-of-the-art natural language processing.

[2] Wolf T., Debut L., Sanh V. (2019). Huggingface’s transformers: state-of-the-art natural language processin. Huggingface’s transformers: state-of-the-art natural language processing. https://arxiv.org/abs/1910.03771.

[3] Gu Y., Tinn R., Cheng H. (2021). Domain-specific language model pretraining for biomedical natural language processing. *ACM Transactions on Computing for Healthcare*.

[4] Pei J., Zhong K., Li J., Xu J., Wang X. (2021). ECNN: evaluating a cluster-neural network model for city innovation capability. *Neural Computing & Applications*.

[5] Guo J., He H., He T. (2020). GluonCV and GluonNLP: deep learning in computer vision and natural language processing. *Journal of Machine Learning Research*.

[6] Yadav V., Bethard S., Sharp R. (2019). A survey on recent advances in named entity recognition from deep learning models. https://arxiv.org/abs/1910.11470.

[7] Akbik A., Bergmann T., Vollgraf R. Pooled contextualized embeddings for named entity recognition.

[8] Al-Moslmi T., Ocana G. M., Opdahl L. A. (2020). Named entity extraction for knowledge graphs: a literature overview. *IEEE Access*.

[9] Priyadharshini R., Chakravarthi B. R., Vegupatti M., McCrae J. P. Named entity recognition for code-mixed Indian corpus using meta embedding.

[10] Luo Y., Xiao F., Zhao H. Hierarchical contextualized representation for named entity recognition.

[11] Pearson C., Seliya N., Dave R. (2021). Named entity recognition in unstructured medical text documents. https://arxiv.org/abs/2110.15732.

[12] Zhao S., Liu T., Zhao S., Wang F. (2019). A neural multi-task learning framework to jointly model medical named entity recognition and normalization. *AAAI Conference on Artificial Intelligence*.

[13] Bhatia P., Celikkaya B., Khalilia M. Comprehend medical: a named entity recognition and relationship extraction web service.

[14] Xiao Y., Zhao Q., Li J., Chen J., Cheng Z. MLNER: exploiting multi-source lexicon information fusion for named entity recognition in Chinese medical text.

[15] Zhang M, Wang J, Zhang X Using a pre-trained language model for medical named entity extraction in chinese clinic text.

[16] Friedman C., Alderson P. O., Austin J. H. M., Cimino J. J., Johnson S. B. (1994). A general natural-language text processor for clinical radiology. *Journal of the American Medical Informatics Association*.

[17] Wu S. T., Liu H., Li D. (2012). Unified medical language system term occurrences in clinical notes: a large-scale corpus analysis. *Journal of the American Medical Informatics Association*.

[18] De Bruijn B., Cherry C., Kiritchenko S., Martin J., Zhu X. (2011). Machine-learned solutions for three stages of clinical information extraction. *Journal of the American Medical Informatics Association*.

[19] Roberts K., Harabagiu S. M. (2011). A flexible framework for deriving assertions from electronic medical records. *Journal of the American Medical Informatics Association*.

[20] Torii M., Wagholikar K., Liu H. (2011). Using machine learning for concept extraction on clinical documents from multiple data sources. *Journal of the American Medical Informatics Association*.

[21] Clark C., Aberdeen J., Coarr M., Kirsch D. T., Wellner B., Yeh A., Hirschman L. (2011). MITRE system for clinical assertion status classification. *Journal of the American Medical Informatics Association*.

[22] Luo L., Yang Z., Yang P. (2018). An attention-based bilstm-crf approach to document level chemical named entity recognition. *Bioinformatics*.

[23] Peters M. E., Ammar W., Bhagavatula C., Power R. (2017). Semi-Supervised Sequence Tagging with Bidirectional Language Models. *Annual Meeting of the Association for Computational Linguistics*.

[24] Ouyang E., Li Y., Jin L. Exploring n-gram character presentation in bidirectional rnn-crf for chinese clinical named entity recognition.

[25] Dong X., Chowdhury S., Qian L., Guan Y., Yang J., Yu Q. Transfer Bi-directional LSTM RNN for named entity recognition in Chinese electronic medical records.

[26] Wu Y., Jiang M., Lei J. (2015). Named entity recognition in Chinese clinical text using deep neural network. *Studies in Health Technology and Informatics*.

[27] Unanue I. J., Borzeshi E. Z., Piccardi M. (2017). Recurrent neural networks with specialized word embeddings for health-domain named-entity recognition. *Journal of Biomedical Informatics*.

[28] Zhang J., Li J., Wang S. Category multi-representation: aunified solution for named entity recognition in clinical texts.

[29] Cai X., Dong S., Hu J. (2019). A deep learning model incorporating part of speech and self-matching attention for named entity recognition of Chinese electronic medical records. *BMC Medical Informatics and Decision Making*.

[30] Zhang Z., Zhou T., Zhang Y., Pang Y. (2019). Attention-based deep residual learning network for entity relation extraction in Chinese emrs. *BMC Medical Informatics and Decision Making*.

[31] Lu N., Zheng J., Wu W., Yang Y., Chen K., Hu W. Chinese clinical named entity recognition with word-level information incorporating dictionaries.

[32] Chen A., Peng F., Shan S. Chinese named entity recognition with conditional probabilistic models.

[33] Zhou J., Qu W., Zhang F. (2013). Chinese named entity recognition via joint identification and categorization. *Chinese Journal of Electronics*.

[34] Yang F., Zhang J., Liu G. (2018). *Five-Stroke Based Cnn-Birnn-Crf Network for Chinese Named Entity Recognition*.

[35] Ding R., Xie P., Zhang X., Lu W., Li L., Si L. (2019). Neural multi-digraph model for chinese ner with gazetteers. *Annual Meeting of the Association for Computational Linguistics*.

